The article "Design and Implementation of Obstetric Central Monitoring System Based on Medical Image Segmentation Algorithm" was published in 2022. Journal: J Healthc Eng.

# Design and Implementation of Obstetric Central Monitoring System Based on Medical Image Segmentation Algorithm

**DOI:** 10.1155/2022/3545831

**Published:** 2022-04-28

**Authors:** Yuanyuan Zhang, Hua Nie

**Affiliations:** ^1^Department of Gynecology and Obstetrics, Hanyang Hospital, Wuhan University of Science and Technology, Wuhan, Hubei 430053, China; ^2^Obstetrics and Gynecology of Wuchang Hospital, Wuhan, Hubei 430063, China

## Abstract

At present, the incidence of emergencies in obstetric care environment is gradually increasing, and different obstetric wards often have a variety of situations. Therefore, it can provide great help in clinical medicine to give early warning and plan coping plans according to different situations. This paper studied an obstetrics central surveillance system based on a medical image segmentation algorithm. Images obtained by central obstetrics monitoring are segmented, magnified in detail, and image features are extracted, collated, and trained. The normal distribution rule is used to classify the features, which are included in the feature library of the obstetric central monitoring system. In the gray space of the medical image, the statistical distribution of gray features of the medical image is described by the mixture model of Rayleigh distribution and Gaussian distribution. In the gray space of the medical image, Taylor series expansion is used to describe the linear geometric structure of medicine. The eigenvalues of Hessian matrix are introduced to obtain high-order multiscale features of medicine. The multiscale feature energy function is introduced into Markov random energy objective function to realize medical image segmentation. Compared with other segmentation algorithms, the accuracy and sensitivity of the proposed algorithm are 87.98% and 86.58%, respectively, which can clearly segment small medical features.

## 1. Introduction

More and more scholars propose a variety of feature machine vision detection algorithms to achieve feature classification, width measurement, and feature stitching. At present, feature region segmentation algorithms are mainly based on threshold, edge detection operator, and deep learning. In the feature image segmentation algorithm based on threshold, due to the lack of considering the noise of different factors such as illumination, debris, texture, and stains of the feature image, the feature segmentation effect of the algorithm is poor and unstable under complex background conditions, and the generalization ability and robustness of the algorithm are low.

In the image feature detail retrieval, Yang uses the Hessian matrix to enhance and denoise the image and then selects the valley value near the peak of the gray histogram of the feature image as the image segmentation threshold. Although it is difficult to determine the valley value for a simple image, the segmentation result is easy to lose the feature details [1]. Akagic et al. propose an improved PCNN image segmentation method based on the analysis of the corresponding relationship between the dynamic threshold and the mean value of the pulse output mapping region. The algorithm has good segmentation performance for the image with mixed gray levels. However, for the feature image with both dark and bright targets, the segmentation results are prone to feature miss detection, and for the subtle part of feature extension, the segmentation results are not accurate, segmentation results are prone to fracture, and segmentation performance is poor in complex images [2]. Wang Q proposed edge detection algorithms using Laplace, Sobel, Prewitt, Roberts, and canny operators to realize automatic feature detection. These edge operator-based feature detection algorithms only detect the edge information of features due to noise sensitivity and cannot identify the width data of features, so they cannot provide scientific basis for judging the degree of pavement damage [3]. Krizhevsky at al. introduce anisotropy measure into feature detection. Small measurement scale is easy to cause feature fracture, while large measurement scale leads to feature false detection. Due to complex feature structure, different widths, and other features, the algorithm cannot meet the requirements of feature detection with different widths [4]. Hoang et al. introduce a variety of image denoising and enhancement algorithms to the empirical canny operator to segment and extract feature information. The algorithm has good segmentation performance for the feature image with shadow. Because the canny operator can only select a fixed segmentation threshold, it is easy to lose the pixels in the feature for a wide range of features, resulting in unsatisfactory segmentation effect [5].

In medical image segmentation feature optimization, Ying et al. propose a feature segmentation algorithm based on support vector machine, which uses greedy intelligent search to optimize canny operator's image segmentation threshold. The selection of ideal threshold directly determines the image segmentation effect. For complex scenes, the segmentation effect of this algorithm is poor [6]. Yoo and Kim introduce full convolution network based on encoder-decoder network architecture into image feature detection, select u-net network structure as the decoder, integrate high-level and low-level features, and expand network depth to complete feature details' recovery. Therefore, feature detection ability and accuracy are improved, but the speed and real-time performance of feature detection need to be further improved [7]. Li proposed a convolutional neural network feature detection method. Firstly, the convolutional neural network was trained by using the created feature image set; then, the feature classification was completed based on the generating model, and finally, the feature was extracted. Because the algorithm only has good processing effect on the feature image with simple background, it has a small scope of application and poor portability and replaceability [8]. Wang Sen proposed a feature detection method based on convolution neural network, which uses 4-layer convolution neural network to complete feature extraction of the feature block image [9]. The above research mostly uses the road feature segmentation algorithm based on deep learning and uses the fitting function of neural network to achieve feature segmentation. However, the parameter setting of multilayer network training in the deep learning model of feature detection easily leads to overfitting phenomenon, and the calculation is time-consuming and complex.

This paper studies the obstetric central monitoring system based on medical image segmentation algorithm and proposes an obstetric medical image segmentation algorithm which combines high-order multiscale features. In this paper, the image obtained by obstetric central monitoring is segmented, the details are enlarged, and the image features are extracted, matched, and learned. Normal distribution rules are used to classify the functions contained in the functional library of the central obstetrics monitoring system. In the gray space of a medical image, the statistical distribution of the gray features of the medical image is described by a mixed model of the Rayleigh distribution and Gaussian distribution. In the gray space of medical images, Taylor series expansion is used to describe the linear geometric structure of medicine. The eigenvalues of Hessian matrix are introduced to obtain high-order multiscale features of medicine. The multiscale feature energy function is introduced into Markov random energy objective function to realize medical image segmentation.

## 2. Experiment and Method

### 2.1. Research Content

In order to solve the problem of poor segmentation effect of the above image segmentation algorithm with complex background features, this paper proposes a feature image segmentation algorithm combining high-order multiscale features. Observed feature images fall into two categories: background and feature. Feature backgrounds and targets are modeled by Rayleigh and Gaussian distributions, Taylor series expansions are introduced to describe the gradient direction of features, and higher-order multiscale features of feature images are constructed by scale transformation. Multiscale function and gray likelihood energy function are introduced at Markov random field. The conditional iterative algorithm is used to estimate the maximum a posteriori probability of feature label field to realize feature image segmentation.

### 2.2. Medical Target Detection

In the field of medicine, image target detection is a necessary condition for diagnosis and treatment. Abnormal positions such as lesions can be detected with the output probability of the discriminant model. In this paper, we combine guns with high-speed r-CNN to detect images. This improves detection efficiency and allows the computer to achieve unsupervised “detection” of the combination of gun and fully convolutional network (FCN). Using DCGANs for image detection, the model can effectively improve the accuracy of detection:

(1) $$\begin{array}{c} {\text{GANs}}_{j}=\sum_{j=1}^{N}X_{ij},\\ P_{ij}=\frac{X_{ij}}{X_{j}}v_{i}^{T}v_{j}+b_{i}+b_{j}. \end{array}$$

Enhanced semisupervised GANs for detection of diabetic retinopathy has achieved a higher detection accuracy *J* and generalization ability of *F*:

(2) $$\begin{array}{c} J=\sum_{i,j}^{N}f\left(X_{ij}\right){\left(v_{i}^{T}v_{j}+b_{i}+b_{j}-\log\left(X_{ij}\right)\right)}^{2},\\ F\left(\log\left(X_{ij}\right)\right)=\frac{{\left\|\log\left(X_{ij}\right)\right\|}^{2}}{1+{\left\|\log\left(X_{ij}\right)\right\|}^{2}}\frac{\log\left(X_{ij}\right)}{\left\|\log\left(X_{ij}\right)\right\|}. \end{array}$$

The AnoGANs model can quickly detect unsupervised anomalies, and the model has high accuracy:

(3) $$\begin{array}{c} \lambda \left(Ai,Aj\right)=\left[\log\left(\frac{\left|x_{A_{i}}-a_{A_{j}}\right|}{w_{A_{j}}}\right),\;\log\left(\frac{\left|y_{A_{i}}-y_{A_{j}}\right|}{h_{A_{j}}}\right),\;\log\left(\frac{w_{A_{i}}}{w_{A_{j}}}\right),\;\log\left(\frac{h_{A_{i}}}{h_{A_{j}}}\right)\right],\\ c_{ij}=\frac{e^{b_{ij}}+v_{i}^{T}v_{j}+b_{i}+b_{j}}{\sum_{k}e^{b_{ik}}}. \end{array}$$

Using GANs to detect hard exudation of color fundus images, the average sensitivity of e-ophtha-EX and DIARETDB1 datasets has been improved. The CGANs model is used to detect glaucoma automatically, and good results are obtained:

(4) $$\begin{array}{c} v_{t}=\frac{\left(w_{1}^{1},w_{2}^{1},w_{3}^{1},w_{4}^{1},w_{5}^{1}\right)}{v_{i}^{T}v_{j}+b_{i}+b_{j}}. \end{array}$$

In this paper, an automatic encoder GANs (agans) is proposed to detect the tumor in the mammogram:

(5) $$\begin{array}{c} v_{j}=\frac{\text{squash}\left(s_{j}\right)}{\sum_{s=1}^{n}{\left(x_{ik}\left(\varepsilon \right)-x_{jl}\left(\varepsilon \right)\right)}^{2}\Delta_{ikjl}\left(\varepsilon \right)},\\ R_{i}=\frac{MI_{i}\left(a\right)-MI_{i}\left(b\right)}{MI_{i}\left(b\right)}. \end{array}$$

This paper proposes an approach to detect fundus diseases based on attention coder and multibranch structure of GANs (AMD GANs). The model has good detection performance for the lesion area. The exponential form of message importance measure (MIM) is used to replace the logarithm form of the original GANs, which achieves good performance in anomaly detection. The algorithm of the generating confrontation model in image target detection C is as follows:

(6) $$\begin{array}{c} C_{ij}=b_{ij}+u_{\left(j|i\right)}v_{j},\\ V_{ikjl}=\left\{\begin{array}{cc} \frac{n}{\Delta_{ikjl}}\sqrt{\sum_{s=1}^{n}{\left(x_{ik}\left(\varepsilon \right)-x_{jl}\left(\varepsilon \right)\right)}^{2}\Delta_{ikjl}\left(\varepsilon \right)}, & \Delta_{ikjl}>0,\\ 0, & \Delta_{ikjl}<0. \end{array}\right) \end{array}$$

### 2.3. Establishment of the Statistical Model

In the process of feature detection, the feature image contains two parts: feature and background. The background part includes low and medium gray areas. The background is modeled by one Rayleigh distribution and two normal distributions. Normal distribution is used to model the characteristic target [10]. For feature images,

(7) $$\begin{array}{c} \cos\left(S,B\right)=\frac{B\cdot S}{\left|B\right|*\left|S\right|}, \end{array}$$

where *S* is the *i*th pixel gray value and *B* is the total number of pixels:

(8) $$\begin{array}{c} B_{t1}\left[i\right]=\sum_{j}\cos\left(w_{i}^{1},w_{j}^{2}\right),\\ W_{t1}=\text{SoftMax}\left(k_{t1}\right), \end{array}$$

where the parameter *W* is the weight coefficient, and the constraint condition is that the parameter *W* is the weight coefficient, and the constraint condition is

(9) $$\begin{array}{c} W=\frac{n\sum_{i=1}^{n}\sum_{j=1}^{n}w_{ij}\left(x_{i}-x\right)\left(x_{j}-x\right)}{\left(\sum_{i=1}^{n}\sum_{j=1}^{n}w_{ij}\right)\sum_{j=1}^{n}{\left(x_{i}-x\right)}^{2}}. \end{array}$$

In the feature image blending model, the parameter set *U* of the gray blending model of the feature image is

(10) $$\begin{array}{c} U=\frac{n\left(x_{i}-x\right)\sum_{j=1}^{n}w_{ij}\left(x_{j}-x\right)}{\sum_{i=1}^{n}{\left(x_{i}-x\right)}^{2}}. \end{array}$$

According to equations (10) and (11), the likelihood function of the gray feature mixture model of the road feature image is described as follows:

(11) $$\begin{array}{c} u_{\left(j|i\right)}=\frac{w_{ij}A_{i}}{\sum_{j=1}^{n}w_{ij}\left(x_{j}-x\right)}, \end{array}$$

(12) $$\begin{array}{c} s_{j}=\sum_{i}c_{ij}u_{\left(j|i\right)}. \end{array}$$

Then, the gray feature model of the feature image is obtained. According to equation (12), the expected likelihood function of the gray feature model of the feature image is established:

(13) $$\begin{array}{c} \mathrm{Pr}=\frac{T}{T+F}, \end{array}$$

where

(14) $$\begin{array}{c} T=\frac{P+N}{P+T+P*+F*}. \end{array}$$

*M* is the number of components of the mixed model, and *N* is the number of pixels of the feature image. It is necessary to process all the pixels of the feature image and speed up the operation speed by multiplying each gray value with the histogram frequency and summating all the gray levels of the feature image:

(15) $$\begin{array}{c} h_{t}=\frac{z_{t}\Theta h_{\left(t-1\right)}}{P+N}+\left(1-z_{t}\right)\Theta h_{t}, \end{array}$$

where *h* is the maximum gray level in volume data and *h*_*t*_ is the frequency of the gray level *t* in histogram. Taking equation (15) into the energy equation in equation (14), the partial derivative of the parameter is calculated and made equal to zero, and the parameter updating formula is obtained:

(16) $$\begin{array}{c} r_{t}=\sigma \left(w_{r}x_{t}+u_{r}h_{t-1}+b_{r}\right),\\ h_{t}=\tan h\left(w_{c}x_{t}+u_{c}\left(r_{t}\Theta h_{t-1}\right)+b_{c}\right). \end{array}$$

So far, the optimization of the feature gray feature hybrid model is completed.

### 2.4. Multiscale Feature Extraction

In the feature image, the whole feature is the tree structure, and the local feature is a linear or block structure. To increase the contrast of features, subtle features and surrounding features are preserved and nonfeature pixels are suppressed. A measurement scale within a specific range is introduced to analyze the local characteristics of the feature image. The Taylor expansion of feature image I in the neighborhood of point *x* is described as follows:

(17) $$\begin{array}{c} XI_{i}=\sum_{j=1}^{n}X_{ij},\;\left(i\neq j\right), \end{array}$$

where *x* is the scale of the image. Based on the theory of image scale space, the second-order directional derivative of the image on scale is calculated by convolution of the Gaussian function and the image:

(18) $$\begin{array}{c} W_{0tikjl}=\sum_{\delta =1}^{n}\Delta_{ikjl}\left(W_{0}\cdot h_{t}\right). \end{array}$$

When the pixel is the feature, the similarity measure function of the image is described as follows:

(19) $$\begin{array}{c} W=\left\{\left(cx_{1},xy_{1},st_{1},et_{1}\right),\left(cx_{n},xy_{n},st_{n},et_{n}\right)\right\}. \end{array}$$

Then, *Y* represents a mapping from the pixel set *s* to the marker set *L*. Therefore, the problem of image segmentation can be solved by calculating the posterior probability *p* (*Y* |*x*) under the observed gray value *X*:

(20) $$\begin{array}{c} P\left(y|x_{t}\right)=\frac{1}{M\left(-r_{t}\right)}. \end{array}$$

It is the likelihood probability of the feature of the feature image, which represents the mapping probability of the feature value of the feature image to the feature mark. The larger the value is, the more appropriate the label is assigned [11]. Taking the negative logarithm of equation (20), the likelihood energy function *U*(*x* |*y*) and the prior energy function *U*(*y*) are defined as

(21) $$\begin{array}{c} \frac{R_{t}}{U\left(x|y\right)}={\left(1+\frac{r_{t}}{\beta }\right)}^{\alpha }. \end{array}$$

In the process of feature image detection, coarse features are easy to segment because of high brightness in the image, while small features and peripheral features are fuzzy and low contrast, which makes feature segmentation very difficult. Therefore, single gray information cannot be effectively segmented, and it is usually necessary to introduce additional feature information to overcome the above problems, the multiscale feature information is introduced into the energy function, and the isotropic MLL model is selected as the Markov random model for feature image segmentation:

(22) $$\begin{array}{c} \text{MLL}\left(y_{t}\right)=\sigma \left(W_{0}\cdot h_{t}\right). \end{array}$$

### 2.5. Segmentation Algorithm Flow

According to the minimum criterion of energy function, the ICM method is used to estimate the label field of features, calculate the parameters of the gray mixed model of the feature image, construct the gray statistical model, and establish the gray features of the feature image [12]. The spatial scale factor is initialized and the quadratic derivative of the feature image is obtained according to the quadratic Taylor expansion of the image. The measurement response value in the multiscale factor is calculated repeatedly. The performance test of the proposed algorithm is completed through the performance test experiment and the comparative analysis experiment of different algorithms. The experimental test samples are provided by Guangxi Academy of Transportation Sciences Co., Ltd, the hardware platform of the experimental environment is Intel (*R*) core (TM) i57200 CPU@2.50 GHz processor, the operating system platform is windows l064 bit system, and the programming software is matlab r2010b. The graphic segmentation framework of the obstetric central monitoring system is shown in Figure 1.

Update the random weights of the features to obtain the parameters of the hybrid model, minimize the labeling field of the scalar energy function, and judge the current number of iterations. If the current number of iterations is equal to the maximum number of iterations, the algorithm ends [13].

## 3. Results

### 3.1. Scale Analysis of Medical Image Segmentation Network

The RMSE of the proposed feature gray model obtains the optimal solution of the parameter Θ in a short number of iterations. When the number of iterations is small, the error of the statistical model presents a slight disturbance and the disturbance is small, but with the increase of the number of iterations, the convergence speed of the proposed algorithm is faster. The convergence curve shows that the algorithm has stable optimization and powerful model parameter optimization. At the same time, the final feature image is determined based on the characteristics of the feature image and the EM algorithm. This allows the gray model to more accurately simulate the histogram distribution of the feature image.

As shown in Figure 2, the fine prediction of large-scale targets in medical image segmentation network is more likely to cause the problem of small-scale target missing and rough category boundary. In view of the shortcomings of medical image segmentation network, its spatial modeling ability is improved to capture richer context information, and the boundary problem is optimized [14]. The improved hierarchical medical image segmentation network takes ResNet-101 as the backbone network, which includes three parts: encoder, decoder, and optimizer.

As shown in Table 1, medical image segmentation network takes the V3 model as the encoder and continues to use the original expansion convolution of the V3 model ASPP module with expansion rates of 6, 12, and 18. With the continuous extraction of image feature information by convolution neural network, the resolution of feature image is decreasing. When extracting low-resolution features, expanded convolution can better capture the details of small- and medium-sized targets in the image. At the same time, if you want to segment large targets, you need to get greater sensitivity. Compared with the expansion convolution with expansion rate of 18, the expansion convolution with expansion rate of 24 has a greater sensitivity, which is more advantageous in segmenting large-scale targets. Comparing the ASPP parameters proposed in this paper with the ASPP modules (6, 12, 18) provided by the V3 + model, the effect of the parameters proposed in this paper is better than the original parameters, so we use 4, 8, 12, and 24 to replace the expansion convolution expansion rate in the original ASPP module [15].

As shown in Figure 3, the larger the Miou value is, the more accurate the predicted segmentation graph is. During the experiment, ResNet-101 was selected as the backbone network [16]. The batch size is set to 8 and data expansion is used. The Pascal VOC 2012 extended dataset adjusts the resolution of the input image to 400*∗*400, randomly scales the image within range, and then randomly crops the image to 380*∗*380 for training. In the cityscape dataset, the resolution of the input image is adjusted to 768*∗*768, the image is randomly scaled within the range, and the image is randomly cropped to 512*∗*512 size for training. The processed samples are more random, which can more effectively prevent the overfitting problem in the training process [17].

As shown in Figure 4, it can obtain greater sensitivity without increasing parameter complexity. Therefore, when multiscale feature extraction is carried out, selecting the appropriate expansion rate can obtain image feature information more effectively [18]. It can be seen from the prediction results that, in the first line of the test image, the medical image segmentation network can segment large-scale objects (aircraft) quite clearly, but it has obvious defects in the segmentation of small-scale objects with occlusion; through comparison, it can be seen that the medical image segmentation network using FReLU activation function for precision compensation has better semantic capture ability for small-scale targets as a whole [19]. In the second line of the test image, the medical image segmentation network predictions have a fuzzy segmentation target boundary and misrecognition issues within the target class. By comparison, it can be seen that the prediction results of the medical image segmentation network using the FReLU activation function for accuracy correction have high boundary accuracy and can effectively reduce the problem of misrecognition in the class [20].

As shown in Figure 5, the medical image segmentation network using ResNet-101 as the pretraining model and the improved ASPP module is used as the baseline. The original nonlinear activation function ReLU in the network is replaced by the visual activation function FReLU, and the data is expanded in PASCAL VOC 2012 before and after improvement. Compared with the original medical image segmentation network, the result of the set comparison is improved by 0.009, and the segmentation accuracy of most objects is improved by 0.009, which proves the effectiveness of the FReLU activation function for network optimization.

The visualization effect of the improved algorithm on cityscapes dataset is shown in Figure 6. Compared with the red marked area, the first line of prediction results still show that the prediction accuracy of medical image segmentation network for small- and medium-sized yellow traffic signs in the image is low, and the prediction of vehicle boundary is rough and there are large errors; by extracting more abundant spatial context information, the proposed algorithm has stronger prediction ability for small-scale yellow traffic signs in the image and optimizes the object boundary. As can be seen from the second line of prediction results, the medical image segmentation network mistakenly identifies a large number of sky scenes in the image as wall parts due to the intersection of sky scenes and wall parts. The algorithm used in this paper can more accurately identify the boundary contour of sky and wall by accurately dividing the boundaries of various categories, to avoid the classification confusion between adjacent categories [21].

At the same time, under the same experimental equipment and superparameter settings, on cityscapes' dataset, the algorithm is compared with the classical algorithm and the latest related research algorithm. The comparative experimental results are shown in Table 2. We find that the algorithms in this paper give better segmentation results in various categories such as buildings and walls. From the third line of the prediction results, we can see that the medical image segmentation network cannot predict the terrain category on the left and incorrectly recognizes the terrain area on the right as a sidewalk. The algorithm proposed in this paper corrects the problem of mistakenly recognizing the truck and the right terrain, effectively predicts the unrecognized terrain in medical image segmentation, and makes the prediction results more precise [22]. The experimental results show that the proposed algorithm can improve the original medical image segmentation network in small-scale prediction and in class error recognition and fuzzy boundary.

Set the same parameters of the ladder network and the baseline network, and test in cityscapes' dataset. The Miou values of each category before and after the improvement are shown in Figure 7. By comparison, it can be seen that compared with the original medical image segmentation network model, the overall Miou value of the improved network is improved by 0.013, and the Miou values of each category are improved to varying degrees.

### 3.2. Fusion Effect Analysis of Segmented Image

As shown in Table 3, the original medical image segmentation model only designs a simple decoder, which mainly deals with the fusion operation of high-level and low-level feature images. In the feature map, cross-layer fusion, a 1/4x downsampling feature map of the ResNet-101 network, contains a wealth of low-level spatial information, and a 1/16 feature map generated by the encoder ASPP module contains a wealth of high levels. Consider that it contains semantic information. Upsample the feature map generated by the encoder ASPP module four times because the size of the high-level feature map generated by the ASPP module needs to be adjusted to the size of the low-level feature map generated by the backbone network. Then, merge with the quarter feature map generated by the backbone network.

As shown in Figure 8, the 1/16 feature map generated by the backbone network is convoluted in parallel, and six 1/16 feature maps with 256 channels are generated. Splice the 6 feature maps in the channel dimension to generate an ASPP module feature map. This allows you to better extract features of multiscale images and improve the segmentation capabilities of networks of various scale objects. As an important part of the encoder, it is still used in the field of medical image segmentation due to its excellent performance in multiscale feature extraction.

Smaller expansion rate can segment small-scale targets more effectively. Larger expansion rate is more effective in segmentation of large targets. The ASPP module of the encoder is improved. In deep learning, convolutional neural network has good performance superiority in processing visual tasks. Nonlinear activation function is a necessary part of convolutional neural network to provide good nonlinear modeling ability. At present, the common activation functions are ReLU and its evolved PReLU.

As shown in Figure 9, the funnel condition is a square sliding window with preset parameters, which is realized by depth separable convolution and data normalization (BN), which can improve the spatial dependence between pixels, activate the spatial insensitive information, obtain rich spatial context information, and improve the pixel-level spatial modeling ability. Only a few parameters and a little complexity are introduced. In addition to the vertical and horizontal directions, oblique lines and arcs are also common in natural objects. The pixel space information extracted by different activation layers is represented by squares of different sizes. The oblique lines and arcs' activation domain is constructed by limit approximation thinking, so as to avoid the lack of modeling ability caused by only using the normal horizontal and vertical activation domain.

As shown in Figure 10, in the direction branching, we also use the 1 × 1 convolution, BN normalization, and ReLU activation function to generate 256 channel number feature map and then use the linear classifier composed of 1 × 1 convolution for upsampling prediction. Considering that the discrete partition performs better than the conventional continuous direction map, the whole direction of the ground real scene map is evenly divided into eight discrete partitions. The generated discrete pattern contains orientation information for each boundary pixel and a different pixel, and the generated discrete pattern is globally multiplied by a binary boundary pattern consisting of 0s and 1s. The orientation of the boundary pixel represented by the value 1 is treated as follows. The internal pixel area, which does not change but is represented by a value of 0, is not included in the calculation. The inner pixel with 0 value in the boundary image is retained and the direction vector in the direction image corresponding to the boundary pixel with 1 value is extracted. The boundary image and the direction image are fused into an offset image with different direction offset information of each boundary pixel, and the boundary pixels are adjusted through the optimization formula.

As shown in Figure 11, when the Gaussian noise variance is greater than 0.06, the segmentation error of the proposed algorithm increases slowly, showing good robustness. When the spatial scale matches the medical width, the medical measurement response value is maximized and the maximum response value is treated as an extended medical measurement. At various scales, the algorithm can enhance the medical structure of each scale. Due to the difference in scale and the strong randomness of the medical structure, it is not possible to obtain the medical response value of each scale on one scale, which causes a fracture phenomenon. At the same time, the adjacent medicine interferes with each other, and the two medicines are detected as one, especially when the scale factor is large. The medical similarity measure function has a uniform response in the medical area, and both fine medicine and peripheral medicine are enhanced, and the structure of nonmedical organizations is suppressed.

As shown in Figure 12, the proposed algorithm is verified by various typical medical images. Compared with other segmentation algorithms, the accuracy of the proposed algorithm is 87.98%, and the sensitivity is 86.58%, which can clearly segment small medical features. The previous test results verify the feasibility of the proposed algorithm for obstetric medicine segmentation operation, but it does not reflect the unique advantages of this segmentation algorithm. All the algorithms can complete medical segmentation for medical objects, but the effect is quite different. K-means algorithm only relies on the gray level of the medical image to complete the medical image segmentation by clustering, so the segmentation result of this algorithm is poor. In this algorithm, the multidistribution gray limited mixed model is adopted, and the high-order multiscale features of the image are fused. The local characteristics of the medical image are analyzed in a certain range of measurement scale. It can enhance the medical targets and suppress the nonmedical targets. The segmentation results are more detailed, and the medical targets are continuous. It has higher segmentation accuracy than other segmentation algorithms, and it can provide high quality data for medical stitching and width measurement.

## 4. Discussion

Through a large number of experiments, the generalization and matching fitness of FReLU function are better than ReLU function. For example, in ImageNet 2012, compared with other effective activation functions, the error rate of top-1 of FReLU activation function in ResNet-50 is only 22.4 on the premise that other parameters remain unchanged. Compared with ReLU, the accuracy was improved by 1.6% and 1.3%, respectively. In ResNet-101, FReLU also performs better than ReLU activation function. With the deepening of network layers, the resolution of input feature map will gradually decrease due to downsampling and spatial pooling operations. Given that the FReLU activation function introduces a small amount of functional complexity and slightly increases the nonlinear activation cost; the original ReLU activation function has been replaced by the FReLU activation function deep in the network framework. Although there is a slight delay in operation, the ReLU activation function can be used to compensate for the potential loss of accuracy caused by the lack of space-independent information. In the existing medical image network, the error rate of boundary segmentation is higher than that of in class confusion. However, the widely used full join conditional random (CRF) in previous studies has little effect on the prediction result graph of medical image segmentation network, so it can no longer be used as the network boundary optimization algorithm of medical image segmentation. Considering that, in the image segmentation results, intraclass pixel segmentation is more reliable than boundary segmentation [23] and that the medical image segmentation network has good intraclass segmentation accuracy on multiple datasets, it is feasible and effective to map the boundary pixels with high error rate to intraclass pixels for result prediction. Considering that HRNet parallel network can always maintain high-resolution feature performance, it is selected as the optimized branch feature map extraction network [24]. In the boundary optimization module, the obtained feature images are sent to the boundary branch and the direction branch, respectively. In the boundary branch, 1 × 1 convolution is used, respectively, and then, the linear classifier composed of 1 × 1 convolution is used for upsampling prediction. The preset threshold is used for boundary division, and those less than the threshold are divided into the target boundary, but not the internal pixels. The boundary graph containing the probability that each pixel belongs to the boundary pixel is generated, and the binary cross-entropy function is used as the boundary branch loss function. In the generated binary boundary graph, the boundary pixel is represented by 1, and the inner pixel is represented by 0. When predicting objects with thick boundaries, only using threshold division is easy to cause false prediction of internal pixels. In order to solve this problem, all the offsets are rescaled by manually setting the scaling factor to reduce the prediction error caused by false pixels [25].

The collected medical images were cut into 512*∗*512 images to form a medical dataset. A total of 20 medical images with rich information were selected for statistical and quantitative analysis with K-means, MRF, and PCNN algorithms. The sensitivity and specificity of this algorithm are similar to the other three algorithms in numerical performance, but the accuracy index reaches 85.93%, which is 24.38%, 13.69%, and 12.95% higher than K-means, MRF, and PCNN algorithms, respectively. The accuracy of medical detection is more important than sensitivity and specificity, especially the medical missed detection has greater harm; for the engineering application of obstetric medical detection, this algorithm has better detection performance.

Based on the medical image segmentation network, this paper constructs a ladder network framework to retain the original network structure of expansion convolution and codec. By improving the spatial pooling pyramid module, the original nonlinear activation function ReLU is replaced by the better visual activation function FReLU to obtain the accuracy compensation; an optimization branch is added after the decoder to refine the rough prediction graph. Experimental results on public datasets of cityscapes show that the ratio of mean intersections and unions in each category of the improved algorithm has been improved to varying degrees, better capturing small targets and capturing the boundary areas of objects. This indicates that it can be segmented. Convolution and upsampling are then performed to generate a forecast results graph. In the original codec network, the ReLU activation function is used for nonlinear activation. The reliability of the ReLU activation function is recognized in the field of deep learning, but it lacks the ability of pixel-level modeling in computer vision. Therefore, this paper uses the two-dimensional visual activation function FReLU to replace the ReLU activation function in the codec to obtain accuracy compensation. In the aspect of branch optimization, considering that the original network does not use the model algorithm to optimize the generated result graph, the improved medical image segmentation network adds an optimization branch for segmentation results. In the optimization branch, the boundary offset map including each pixel offset is generated by boundary map and direction map, and the generated rough prediction map is adjusted by coordinate mapping. After thinning, the target contour of the prediction map is consistent, the boundary is clear, and the prediction accuracy is higher.

## 5. Conclusions

In this paper, we propose an image segmentation algorithm for obstetrics based on high-order multiscale features. In the gray space of the medical image, the statistical distribution of gray features of the medical image is described by the mixture model of Rayleigh distribution and Gaussian distribution. In the gray space of the medical image, Taylor series expansion is used to describe the linear geometric structure of medicine, and the eigenvalues of the Hessian matrix are introduced to obtain the high-order multiscale features of medicine. Multiscale feature energy function is introduced into Markov random energy objective function to realize medical image segmentation. Medical image segmentation is different from object detection and image classification in computer vision. Specifically, medical image segmentation is to distinguish what the target object is and where the target object is in the image at the pixel level. That is, the targets in the image are first detected, then contoured between each individual and the scene, and finally they are categorized and colored to represent those that belong to the same category. Compared with other segmentation algorithms, the proposed algorithm has an accuracy of 85.93% and a sensitivity of 0.6387%, which can segment small medical images clearly.

## Figures and Tables

**Figure 1:** Graphical segmentation frame of the obstetric central monitoring system.

**Figure 2:** Fine prediction of image large-scale targets.

**Figure 3:** The more accurate predicted segmentation map.

**Figure 4:** Image feature information and expansion rate.

**Figure 5:** Original nonlinear activation function.

**Figure 6:** Visualization on the dataset.

**Figure 7:** Ladder network baseline network parameters.

**Figure 8:** FIG generation backbone network convolution of characteristics.

**Figure 9:** Square sliding window with preset parameters.

**Figure 10:** Ground real scene diagram of the gynecological monitoring system.

**Figure 11:** Fine prediction of Gaussian noise variance target.

**Figure 12:** The efficiency of the algorithm for typical medical images.

**Table 1:** Medical image segmentation network encoder data.

Item	Article mean	Sensitivity	Accuracy	Error rate	Liver segmentation
Admire	3.93	5.77	1.51	2.12	0.11
Feel	4.16	5.12	2.31	4.45	−0.12
Competition	3.4	7.04	2.35	5.41	1.84
Trained	6.4	8.74	1.89	6.91	1.97
Blend	6.56	10.7	3.12	8.57	1.93

**Table 2:** The algorithm in this paper and the classic algorithm.

Item	Accuracy	Error rate	Liver segmentation	Standard deviation	Standard deviation
1	−0.45	5.77	6.09	2.23	1.6
2	1.51	5.75	6.88	1.49	0.7
3	0.81	7.15	7.93	2.21	0.51
4	1.26	8.03	7.42	1.67	1.1
5	1.68	7.47	6.45	0.81	1.57

**Table 3:** The overall network MioU value of the medical image segmentation network model.

Item	Traditional mean	Article mean	Sensitivity	Accuracy	Error rate
1	3.12	4.03	5.2	5.27	5.06
2	1.12	4.12	4.83	5.48	3.96
3	1.42	3.65	5.52	4.01	4.18
4	0.44	4.57	6.26	4.49	3.97
5	0.2	3.28	6.96	2.53	2.92

## Data Availability

Analytical permission from the data provider has not been obtained because of trade confidentiality.
